The article "Observation on the Nursing Effect of the Whole Process in Patients with Severe Intracranial Hemorrhage" was published in 2022. Journal: Comput Math Methods Med.

# Observation on the Nursing Effect of the Whole Process in Patients with Severe Intracranial Hemorrhage

**DOI:** 10.1155/2022/1546019

**Published:** 2022-07-04

**Authors:** Zhongwei Su, Wei Guo, Yun Luo, Yao Wang, Yue Du

**Affiliations:** Emergency Department, Beijing Tiantan Hospital, Capital Medical University, Beijing, China

## Abstract

**Objective:**

The goal of this study was to look at the clinical impact of the entire process of nursing care for patients with severe cerebral hemorrhage.

**Method:**

From January 2018 to December 2019, the clinical data of 160 patients with severe cerebral hemorrhage who were hospitalized to our hospital were reviewed retrospectively. They were separated into two groups based on their admission: routine and complete procedure. The routine group used routine emergency care, the whole process group was provided first aid care with whole process nursing. The diagnosis and treatment time, the success rate of emergency care, the incidence of adverse events, and the complaint rate were compared between the two groups.

**Results:**

The treatment time, emergency examination time, and preoperative rescue time of emergency patients in the whole process group were significantly shorter than those in the conventional group, with statistically significant differences (all *P* < 0.05). The rescue success rate of emergency patients in the whole process group was 95.00% (76/80), and the rescue success rate of emergency patients in the routine group was 83.75% (67/80); the difference was statistically significant (*χ*^2^ = 4.378, *P* = 0.034). The complaint rate of emergency patients in the whole process group was 2.50% (2/80), while that in the routine group was 8.75% (7/80), with statistically significant difference (*χ*^2^ = 4.732, *P* = 0.024). The incidence of total nursing adverse events was 6.25% (5/80) in the whole process group and 17.50% (14/80) in the routine group; the difference was statistically significant (*χ*^2^ = 5.011, *P* = 0.027).

**Conclusion:**

The implementation of whole process nursing care for patients with severe intracranial hemorrhage can shorten the time-consuming first aid for patients with intracranial hemorrhage. And it also can improve the rescue success rate of patients and reduce the incidence of adverse events and complaints, which represents a significant clinical application effect.

## 1. Introduction

Intracranial hemorrhage is a very common disease in clinical neurosurgery. Intracranial hemorrhage is one of the symptoms of “stroke” in traditional Chinese medicine, and most patients had hypertension or cerebrovascular malformation [1–3]. Intracranial hemorrhage is a hemorrhage caused by nontraumatic rupture of blood vessels in the brain parenchyma. The blood clot caused by hemorrhage leads to edema at the bleeding site and compression of cerebral nerves, and the gradual increase in cranial pressure leads to a series of clinical symptoms [4, 5]. Among them, intracranial hemorrhage caused by hypertension is very common. Its early manifestations are vomiting, impaired movement, and difficult walking. The main clinical manifestations are headache, nausea, drowsiness, and so on, and severe diseases such as hemiplegia and speech disorder may occur, even endangering the life of the patients, which has a certain impact on the prognosis of the patients' quality of life [6, 7]. The therapeutic effect of patients with intracranial hemorrhage is closely related to the timeliness of treatment. Due to the lack of early warning of intracranial hemorrhage, people often ignore the importance of the harm of intracranial hemorrhage. In addition, the rapid onset, deterioration, and impact on the body of intracranial hemorrhage are closely related to the time when patients are treated [8, 9]. The recognition of the status of rehabilitation nursing for patients with intracranial hemorrhage is considered “three points of treatment and seven points of nursing” in the medical industry, which shows the importance of efficient nursing for the rehabilitation of patients with intracranial hemorrhage. For patients with severe intracranial hemorrhage, a set of reasonable care should be given early. Intervention measures are urgent. Patients with intracranial hemorrhage have brought great difficulties and challenges to medical staff in the process of treatment and nursing due to their difficult actions, vague speech, and ambiguous language [10]. Whole process nursing is a continuous, full-process, efficient, and zero-distance nursing care method implemented by medical staff to patients. In order to improve the rescue level of critical patients, the whole process nursing was applied in the treatment of patients with severe intracranial hemorrhage in this study, and the effect was good. It is reported as follows.

The paper is organized as follows: the materials and methods are presented in Section 2.  Section 3 discusses the experiments and results.  Section 4 is discussed in combination with the relevant data analysis of this study. Finally, the research work is concluded; it points out the specific sharing made by this research and the future development direction of this field.

## 2. Materials and Methods

### 2.1. Normal Information

The clinical data of 160 patients with severe intracranial hemorrhage admitted to our hospital from January 2018 to December 2019 were retrospectively analyzed. They were divided into the routine group (January-December 2018) and the whole process group (January-December 2019) according to their admission sequence, with 80 patients in each group. There were 56 males and 24 females in the whole process group. The average age was 40.23 ± 5.47 years old; the AIS-ISS injury score ranged from 16 to 50 points, with an average score of 30.52 ± 3.63. There were 58 males and 22 females in the routine group. The average age was 40.15 ± 5.26 years old; the AIS-ISS injury score ranged from 16 to 50 points, with an average score of 31.24 ± 3.81. There was no statistically significant difference in general data between the two groups (*P* > 0.05), which was comparable. Comparative results of clinical data are shown in Table 1.

According to the purpose of the study and the relevant research results of previous scholars, the enrollment criteria and exclusion criteria formulated in this study are as follows:

Enrollment criteria were as follows:

1. Hypertension led to severe intracranial hemorrhage
2. Intracranial hemorrhage was confirmed by imaging examination
3. The patients and their families knew and agreed to participate in this study voluntarily

Exclusion criteria were as follows:

1. Severe intracranial hemorrhage caused by other reasons (including congenital cerebral vascular malformation and severe intracranial hemorrhage caused by trauma)
2. Severe functional insufficiency of other organs
3. Patients who had died prior to medical consultation
4. A history of severe cardiopulmonary dysfunction
5. Cognitive, intellectual, and mental disorders
6. A history of physical disability or dysfunction
7. Patients who gave up treatment on their own during rescue
8. Incomplete data

### 2.2. Methods

#### 2.2.1. Routine Group

Conventional emergency care was adopted, and emergency rescue was carried out according to the rescue procedures of ventilation → dilatation → cardiac pump → control of bleeding → operation [11]. Specifically, it was to keep the airway unobstructed and fully inhale oxygen, establish a venous channel for blood transfusion or infusion as soon as possible, test the heart function to restore the cardiac blood function, and control the bleeding and operate as soon as possible. The nursing staff should perform routine examinations and rescues of patients as directed by the doctor, improve preoperative preparation, monitor the physical symptoms of patients with severe cerebral bleeding, and establish venous access as quickly as feasible during the implementation of rescue. And they cooperated with doctors to carry out targeted multiple examinations (such as chest puncture and abdominal puncture) to prevent traumatic shock. After admission, paramedics assisted necessary examination and followed up routine nursing staff after emergency surgery evaluated the injury.

#### 2.2.2. Whole Process Group

Carry out emergency care with whole process care.

*(1) Setting up a Whole Process Nursing Team*. The whole process nursing team first set up a captain, who was the chief commander in the entire emergency care nursing process; one respiratory nurse was on hand to help respiratory doctors in carrying out medical orders; an executive/circulatory nurse assisted the doctor in managing the patient's respiratory and circulatory system. There was one assistant nurse, who cooperated with the doctor to operate instruments and equipment and was responsible for drug delivery, blood sample collection, and other auxiliary examinations. There was one recording nurse, who was responsible for recording basic patient information, rescue records, doctor's orders, and changes in the patient's condition and responsible for outreach work, timely communication with the laboratory, imaging department, and so on, to ensure full cooperation in emergency care. At the same time, prepare a mobile nurse to cooperate with other posts at any time. The management team provided whole process care throughout the first aid care process. The staffing of the whole process nursing team is shown in Figure 1.

*(2) The Whole Process Nursing Service System*. The whole process nursing service system includes the whole process of service consciousness, the whole process of management, the whole process of professional technology, the whole process of first aid, and the whole process of medical cooperation (Figure 2).

1. The whole process of service consciousness

Organize the study of humanized nursing service concept regularly, change the passive service into active service, and emphasize the importance of active service in the rescue of severe intracranial hemorrhage.

(2) The whole process of management

The management team shall refine the routine rescue procedures and formulate the emergency plan for severe intracranial hemorrhage, and the team leader shall evaluate the implementation rules of detection to ensure the implementation of the rescue procedures.

(3) The whole process of professional technology

Hire nursing staff with rich rescue experience to give regular special lectures to strengthen the professional ability of the nursing team.

(4) The whole process of first aid

Select nurses with strong professional competence for consultation, and the attending nurses assist in the judgment of illness. Once confirmed as severe intracranial hemorrhage, immediately start the whole process of nursing and the completion of emergency care nursing task.

(5) The whole process of medical cooperation

The comprehensive treatment mode was adopted for rescue nursing.

The principle of rescue first and payment later was to assist them to go through the admission procedures, and at the same time, nurses cooperated with the doctors to give first aid. This principle not only saves valuable rescue time, improves the treatment effect, and simplifies the process of patients before admission but also improves the satisfaction of patients' family members.

1. Respiratory care [12]

The suction nurse assisted in cleaning up foreign bodies in the patient's mouth, who was ready to attract and suck sputum at any time, keep the airway open, and closely monitor the patient's breathing state to ensure that the airway was open.

(2) Circular care [13]

Circulation nurses assisted in establishing venous access, correcting electrolyte acid-base balance disorder, maintaining circulating blood volume in the trauma area, and preventing cardiac arrest, hemorrhagic shock, and so on.

(3) Condition observation [14, 15]

The team leader closely monitored the patient's condition while managing the rescue scene, focusing on the patient's state of consciousness. In addition, the implementation of the doctor's advice should be checked in a timely manner to prevent errors made by the nursing staff due to stress. At the same time, mobile nurses are on standby to increase the links or posts in need of help, so as to improve the timeliness of work. The flowchart of the whole process nursing is shown in Figure 3.

### 2.3. Observation Target

1. Time indicators for diagnosis and treatment

This includes patient reception time, emergency examination time, and preoperative rescue time. Attendance time referred to the time from the time the medical staff receives the distress call to the time they arrive at the rescue scene. The time of emergency assessment was defined as the sum of the time spent on routine blood tests, coagulation function, blood matching, virus antibody testing, and imaging testing, among other things. Preoperative rescue time referred to the time from the patient's admission to the emergency operating room.

(2) Success rate of emergency care

If the patient's vital signs remained stable and the patient was safely transferred to the relevant department, the rescue was a success. Rescue success rate (%) = number of successful rescue/total number of people × 100%.

(3) Adverse event incidence and complaint rate

Adverse events mainly included pipe shedding, incorrect execution of medical advice, incomplete drug preparation, accidental injury, and so on.

### 2.4. Statistical Analysis

Using SPSS 21.0 statistical software, measurement data was expressed as *x* ± s, and the *t*-test was used; the count data was expressed as a percentage and as a frequency. The theoretical frequency ≥ 0 and ≤5 count data between groups were corrected and tested. If the theoretical frequency was greater than 5, the count data between groups would be tested by *χ*^2^. *P* < 0.05 or *P* < 0.01 indicated that the difference was statistically significant.

## 3. Results

In this section, comparison of diagnosis and treatment time between the two groups, comparison of the rescue success rate between the two groups, and comparison of the incidence of nursing adverse events and complaint rate between the two groups were discussed in detail.

### 3.1. Comparison of Diagnosis and Treatment Time between the Two Groups

The treatment time, emergency examination time, and preoperative rescue time of emergency patients in the whole process group were significantly shorter than those in the conventional group, with statistically significant differences (all *P* < 0.05). Comparison of diagnosis and treatment time is shown in Table 2.

### 3.2. Comparison of the Rescue Success Rate between the Two Groups

The rescue success rate of emergency patients in the whole process group was 95.00% (76/80), and the rescue success rate of emergency patients in the routine group was 83.75% (67/80); the difference was statistically significant (*χ*^2^ = 4.378, *P* = 0.034). Comparison of the rescue success rate is shown in Table 3.

### 3.3. Comparison of the Incidence of Nursing Adverse Events and Complaint Rate between the Two Groups

The complaint rate of emergency patients in the whole process group was 2.50% (2/80), while that in the routine group was 8.75% (7/80), with statistically significant difference (*χ*^2^ = 4.732, *P* = 0.024). The incidence of total nursing adverse events was 6.25% (5/80) in the whole process group and 17.50% (14/80) in the routine group; the difference was statistically significant (*χ*^2^ = 5.011, *P* = 0.027). Comparison of the incidence of nursing adverse events and complaint rate is shown in Table 4.

## 4. Discussion

Intracranial hemorrhage is a common neurological disease, characterized by acute onset, rapid progression, poor prognosis, and high mortality, which seriously threatens the health and life safety of patients. Craniotomy and targeted minimally invasive bloodletting to reduce intracranial pressure are widely used in patients with severe intracranial hemorrhage [16]. The success of brain resuscitation in patients with severe intracranial hemorrhage, whether there is rebleeding in the brain and whether there are nosocomial-acquired lower respiratory tract infections and other related serious complications, is the key to successful treatment, increased survival rate, and reduced mortality [17, 18]. It can be seen that patients with severe intracranial hemorrhage not only depend on the doctor's diagnosis and treatment strategy but also are closely related to the correct nursing intervention measures [19–21]. The whole process of nursing for patients with severe intracranial hemorrhage in the rescue of the clinical effect reduces complications, and the prevention of rebleeding has obvious effects [22–24].

The findings showed that the whole process group's treatment time, emergency examination time, and preoperative rescue time were much shorter than the traditional group's, with statistically significant differences (all *P* < 0.05). The rescue success rate of emergency patients in the whole process group was 95.00% (76/80), and the rescue success rate of emergency patients in the routine group was 83.75% (67/80); the difference was statistically significant (*χ*^2^ = 4.378, *P* = 0.034). The complaint rate of emergency patients in the whole process group was 2.50% (2/80), while that in the routine group was 8.75% (7/80), with statistically significant difference (*χ*^2^ = 4.732, *P* = 0.024). The incidence of total nursing adverse events was 6.25% (5/80) in the whole process group and 17.50% (14/80) in the routine group; the difference was statistically significant (*χ*^2^ = 5.011, *P* = 0.027).

## 5. Conclusion

To summarize, implementing whole process nursing for patients with severe intracranial hemorrhage can reduce the time it takes for patients to receive first aid, increase the success rate of rescue, decrease the incidence of adverse events and complaints, and have a significant clinical application effect. However, due to the rapid onset of severe intracranial hemorrhage and high degree of harm, how to appease the emotion of the patient's family members in the rescue process is also one of the contents of modern nursing. Patients need long-term continuous care and regular examination after discharge. How to prevent the recurrence of intracranial hemorrhage, slow down the complications and sequelae caused by intracranial hemorrhage, and speed up the rehabilitation process have provided new challenges for patients' families and medical staff.

## Figures and Tables

**Figure 1:** The staffing of the whole process nursing team.

**Figure 2:** The whole process nursing service system.

**Figure 3:** Flowchart of the whole process nursing.

**Table 1:** Comparative results of clinical data.

Groups	Cases	Age	GLS	Intracranial hemorrhage (ml)	Time in ICU (h)	Chronic lung disease (cases)	Operation (cases)
Routine group	80	40.15 ± 5.26	7.15 ± 1.03	32.88 ± 5.03	9.15 ± 2.05	58	67
Whole process group	80	40.23 ± 5.47	7.05 ± 1.21	33.51 ± 3.82	9.39 ± 1.92	60	70
*t*		0.32	0.23	-0.091	-0.35	0.0091	0.093
*P*		0.7446	0.852	0.7105	0.7216	0.9204	0.7582

**Table 2:** Comparison of diagnosis and treatment time.

Groups	Cases	Treatment time	Emergency examination time	Preoperative rescue time
Routine group	80	41.34 ± 4.35	32.09 ± 4.52	71.25 ± 8.13
Whole process group	80	35.75 ± 3.30	21.30 ± 3.05	53.24 ± 5.66
*t*		8.956	18.525	15.912
*P*		<0.001	<0.001	<0.001

**Table 3:** Comparison of the rescue success rate.

Groups	Cases	Rescue success	Rate
Routine group	80	67	83.75%
Whole process group	80	76	95.00%
*χ* ^2^			4.378
*P*			0.034

**Table 4:** Comparison of the incidence of nursing adverse events and complaint rate.

Groups	Cases	Complaint rate	Incidence of nursing adverse events
Routine group	80	8.75%	17.50%
Whole process group	80	2.50%	6.25%
*χ* ^2^		4.732	5.011
*P*		0.024	0.027

## Data Availability

The datasets used during the present study are available from the corresponding author upon reasonable request.
